# Phytosynthesis of Titanium Dioxide Nanoparticles Using King of Bitter *Andrographis paniculata* and Its Embryonic Toxicology Evaluation and Biomedical Potential

**DOI:** 10.1155/2021/6267634

**Published:** 2021-10-07

**Authors:** S. Rajeshkumar, J. Santhoshkumar, Leta Tesfaye Jule, Krishnaraj Ramaswamy

**Affiliations:** ^1^Nanobiomedicine Lab, Department of Pharmacology, Saveetha Dental College and Hospital, SIMATS, Chennai 600077, TN, India; ^2^Department of Physics, College of Natural and Computational Science, Dambi Dollo University, Dambi Dollo, Ethiopia; ^3^Centre for Excellence-Indigenous Knowledge Innovative Technology Transfer and Entrepreneurship, Dambi Dollo University, Dambi Dollo, Ethiopia; ^4^Department of Mechanical Engineering, College of Engineering and Technology, Dambi Dollo University, Dambi Dollo, Ethiopia

## Abstract

Phytosynthesis particles are the efficient activity of biomedical and environmental. In this present study, the green synthesis of titanium dioxide (TiO_2_) nanoparticles using the king of bitter herbal plant *Andrographis paniculata* was synthesized and characterized using XRD, SEM, HRTEM, AFM, and antimicrobial, antioxidant, and antidiabetic activities. The size of the particles HRTEM shows 50 nm, and SEM shows the spherical shape, which reveals the synthesis of TiO_2_ nanoparticles. XRD spectrum shows crystallinity of nanoparticles, and an average size is calculated about 22.97 nm. The phytosynthesis TiO_2_ shows the antioxidant and antidiabetic activities. Similarly, toxicity studies have demonstrated the hatching and viability LD 50 value of TiO_2_ 250 *μ*g/L. The current study's findings suggested that phytosynthesis TiO_2_ using extract of *Andrographis paniculata* exposure to potential hazard factors to biomedical and environmental uses.

## 1. Introduction

Nanotechnology appears as a rapidly growing field of science and technology for manufacturing new materials at the nanoscale level. Nanotechnology has a wide application in various fields such as biology, chemistry, physics, and medicine [1]. Nanomaterials are classified into organic and inorganic materials. Metal and metal oxide nanoparticles have great attention in physical, chemical, biological, medical, optical, mechanical, and engineering sciences. Novel techniques are introduced to examine and manipulate single atoms and molecules [2, 3]. Various physical and chemical methods synthesized metal oxide nanoparticles. Some commonly used methods are nonsputtering, solvothermal, reduction, sol-gel technique, and electrochemical technique. These methods are costly, toxic, high-pressure, high-energy, and potentially hazardous [4–7].

The primary reaction in the biosynthesis of nanoparticles is the reduction/oxidation process because it is a bottom-up approach. The microbial enzyme and the plant phytochemicals in antioxidant or reducing properties are usually responsible for preparing metal and metal oxide nanoparticles [8–10]. Bacteria, fungi, and plant extracts such as neem, *Coriandrum*, *Camellia sinensis*, *Nelumbo lucifera*, *Ocimum sanctum*, and several others are used to achieve the synthesis of nanoparticles by the biological method [11]. The advantages of using plant extract are readily available, safe to handle, and possess abroad viability of metabolites. Terpenoids, flavones, ketones, aldehydes, and amides are the phytochemicals responsible for synthesizing nanoparticles [12, 13]. Titanium dioxide has been extensively used as an environmentally friendly and photocatalyst because of its optical properties, high stability, and nontoxicity [14]. TiO_2_ nanoparticles have been used in cosmetics, pharmaceuticals, and skincare wares to protect the skin from UV rays and whiteness [15]. It is also used in paints, plastics, papers, inks, food colourants, and toothpaste [16, 17]. Miller et al. [18] reported that the TiO_2_ generates reactive oxygen species when exposed to ultraviolet radiation, nanoparticulate TiO_2_ used in antibacterial coatings. Other doped metal and metal oxide particles TiO_2_ as silver, gold, copper [19], ferrous, zinc, cerium, Li/ZnO [20], MgO/La_2_O_3_, and Mg/Zr/Sr mixed oxide are used for chemical and physical syntheses. Unfortunately, most metal and metal oxides show several drawbacks like the time taking process, uncontrolled temperature, and poor reusability [21].

Researchers are currently focusing mainly on the synthesis of nanoparticles using green methods that increase biological effectiveness. The plant species of *Andrographis paniculata*, commonly known as kings of bitters and nilavembu in India, belongs to the Acanthaceae family. The species possess pharmacological properties such as antimicrobial, antioxidant, anti-inflammatory, antiparasitic, antihyperglycemic, hypoglycaemic, and antiallergic [22–24]. Other titanium dioxide nanoparticles underwent optical characterization using the UV-Vis spectrometer, structural characterization using scanning electron microscopy, atomic force microscopy, X-ray diffraction, and antimicrobial, antioxidant, and antidiabetic activities. The zebrafish has become a model organism for the study of human illness in recent decades [25] Zebrafish, being nonmammal, are less related to humans than rats in terms of evolution; despite the drawbacks, zebrafish have become more prevalent in illness research because of their case of handling, low cost, rapid development cycle, fecundity, high genetic resemblance to human, and transparent bodies [26].

## 2. Materials and Methods

### 2.1. Chemical and Plant Materials

Titanium (IV) oxide used in this study was purchased from Merck Darmstadt (Germany). All the reagents were used without further purification. The plant *Andrographis paniculata* leaves were collected from the Vellore area, Tamil Nadu, India.

### 2.2. Preparation of the Leaves Extract

*Andrographis paniculata* leaves were collected, and part of the plants was separated and cleaned with distilled water. Those parts were air dried for 7 days and grinded to fine powder. Then, 1 g was weighed and put into a beaker with 100 ml of distilled water and boiled at 60–70°C for about 10 min. Then, the crude extracts were filtered through Whatman No. 1 filter paper and stored in a refrigerator for further use.

### 2.3. Synthesis of TiO_2_ Nanoparticles

The TiO_2_ NPs synthesis has been done from the previously reported literature [27]. Subsequently, 20 ml of leaves extract was taken, and 80 ml of titanium dioxide was added and kept in a shaker for 1 hour at room temperature. After that, the solution was filtered and dried at 80°C for 12 h and calcined at 500°C for 2 h. Then, the powder was stored for further tests.

### 2.4. Characterization of TiO_2_ Nanoparticles

Crystalline structure and the average crystalline size of the synthesized TiO_2_ NPs were characterized using an X-ray diffractometer using a Scifert diffractometer. Synthesis of TiO_2_ nanoparticles reduce the titanium metal ions in a solution of *Andrographis paniculata* leaves extract to characterize by Perkin Elmer Lambda, UV-Visible spectrophotometer. The surface morphology of the titanium nanoparticles was characterized using SEM and AFM. EDX analysis was carried to confirm the presence of titanium dioxide in the particles and to detect the other elementary compositions of the particles. The TGA analysis was done to know how the biosynthesised titanium dioxide nanoparticles changed physical and chemical properties at room temperature 800°C at 20°C per minute.

### 2.5. Antibacterial and Antifungal Activities of Titanium Dioxide Nanoparticles

The antibacterial activity of the synthesized TiO_2_ nanoparticles was performed by the agar well diffusion method. Fresh colonies of *Bacillus* sp., *E. coli*, and *Salmonella* sp. were spread on Muller-Hinton agar plates. 50 *μ*L of titanium dioxide nanoparticles were filled in the well made in the agar. Then, plates were incubated at 36 ± 1°C for 24 h, and the zone of inhibition was measured [28]. The antifungal activity of synthesized titanium dioxide nanoparticles was tested against the *Candida albicans* cultured on Rose Bengal agar plates added with 50 *μ*L of titanium dioxide nanoparticles by the disc diffusion method [29].

### 2.6. Antioxidant and Antidiabetic Activities of Titanium Dioxide Nanoparticles

The antioxidant activity of synthesized titanium dioxide nanoparticles was determined using the DPPH assay method [30]. *A. paniculata* plant extract and TiO_2_ were screened for the antidiabetic activity. It was estimated using the alpha-amylase assay method [31].

### 2.7. Zebrafish Embryotoxicity

#### 2.7.1. Fish Maintenance and Titanium Dioxide Nanoparticle Exposure

Wild-type zebrafish (*Danio rerio*) were obtained from local vendors, India, and housed in individual tanks and maintained in the condition of temperature (28 ± 2°C), light/dark cycle 14 : 10 h), and pH (6.8–8.5). Fish were fed using commercially available dry blood worms or optimum food two times a day. Zebrafish embryos were collected by crossing one female and three males per breeding tank. Briefly, males and females were physically separated by a transparent block the entire night, which was removed the next morning light cycle to allow reproduction. Viable eggs were collected and rinsed at least three times with freshly prepared E3 medium without methylene blue (5 mM NaCl, 0.17 mM KCl, 0.33 mM CaCl_2_, and 0.33 mM MgSO_4_, pH 7.2–7.3) at 28.5°C. The fertilized eggs were immediately placed in 6, 12, and 24-well culture plates (20 embryos in 2 ml solution/well). Each experimental treatment and control group had three replicates. The stock suspension of titanium dioxide nanoparticles was freshly prepared by directly adding titanium dioxide nanoparticles into the E3 medium and dispersed by sonication (50 W, 40 kHz) for 15 min. The pH of the titanium dioxide nanoparticle added E3 medium is maintained at 7.2-7.3. Healthy fertilized embryos were incubated with titanium dioxide nanoparticles concentration of 0, 50, 100, 150, 200, and 250 *μ*g/L for 24–96 hpf. In nanoparticle-exposed groups, dead embryos were removed from plates every 12 h. All the experimental plates were wrapped in a foil to exclude light and maintained at 28°C.

#### 2.7.2. Zebrafish Embryo Evaluation

During the whole exposure period after fertilization, the embryonic developmental stages of zebrafish embryo were observed under a stereomicroscope. The embryos were exposed to titanium dioxide nanoparticle concentrations (0, 50, 100, 150, 200, and 250 *μ*g/L) for 24–78 hpf. The embryonic mortality and hatching rate were evaluated every 24 h. The endpoints used to survey formative danger included developing life/hatchling mortality and embryo hatching rate. Malformations were described and captured among the embryos and larvae from both the control and treated groups. The photographs of malformed embryos were taken under a stereomicroscope (Optica, Italy Model; T3 15 A, Italy), and the percentage of abnormal embryos was counted for every 24 hours [32].

## 3. Results and Discussion

### 3.1. Visual Observation

Figure 1 shows the before and after synthesized titanium dioxide nanoparticles in the *Andrographis paniculata* extract. The TiO_2_ nanoparticles were added to the *A. paniculata* extract and kept in a shaker for 24 hours at room temperature. We can see the colour change after 24 hours, which shows the synthesis of TiO_2_ nanoparticles in the *A. paniculata* extract. The turbid whitish colour changes conform to the TiO_2_ nanoparticle synthesis.

### 3.2. UV-Vis Spectra Analysis

The optical properties of the synthesized TiO_2_ nanoparticle were studied using UV-Vis spectroscopic analysis, which mainly depends on surface plasmon resonance (SPR), which is used to measure the material adsorption onto the surface of metal nanoparticles [13, 33].  Figure 2 shows the surface plasmon resonance of the TiO_2_ nanoparticles synthesized using *A. paniculata*. The plasmon peak and its width depend on the metal nanoparticles size, the nature of the metal, and the medium dielectric constant. The spectra displayed the characteristic of the SPR band of titanium dioxide nanoparticles at 550 nm, which shows the preliminary confirmation of the TiO_2_ nanoparticles.

### 3.3. Shape and Element Identification of TiO_2_ Nanoparticles

The surface morphology and the size of the TiO_2_ nanoparticles were examined by using scanning electron microscopy.  Figure 3(a) shows the scanning electron microscopy images of TiO_2_ nanoparticles synthesized by the plant extract of *A. paniculata* at different magnifications. It is observed that the synthesized nanoparticles are spherical and tetragonal [34]. The clumped appearance might have been due to the aggregation of TiO_2_. The element composition is further confirmed with energy-dispersive X-ray spectroscopy analysis.  Figure 3(b) shows the EDAX analysis of TiO_2_ NPs by *A. paniculata* which confirmed the grown nanoparticles are composed of titanium and oxygen only. The weight percentage composition of Ti and O is 39.97% and 60.03%, respectively. It shows that there are no other impurities present in the sample [35].

### 3.4. Size and Stability of Titanium Dioxide Nanoparticles

Figure 4(a) shows the transmission electron microscopy images of TiO_2_ nanoparticles synthesized by the plant extract of *A. paniculata*, revealing that the particles are monodisperse and spherical in shape. The sizes of particles in the 50 nm range indicated that the TiO_2_ nanoparticles possessed good crystallinity [36].  Figure 4(b) shows the dynamic light scattering images of TiO_2,_ revealing the zeta potential stability was in −40 mV, indicating the activity and stability of nanoparticles [37].

### 3.5. XRD Analysis of Titanium Dioxide Nanoparticles

The XRD pattern of the As-synthesized TiO_2_ nanoparticles is shown in Figure 5. The peaks of the powder materials are identified to the corresponding (101), (112), (200), (211), (213), (220), and (206) crystal planes. All the diffraction peaks are well defined and can be identified to the TiO_2_ nanoparticles (JCPDS-21-1272). The XRD pattern revealed no distinctive peaks associated with other crystalline forms, indicating that the product is anatase phase-pure. From the peak broadening, the average crystallite size of the As-prepared sample was calculated to be around 22.97 nm [38].

### 3.6. AFM Analysis of Titanium Dioxide Nanoparticles

The surface morphology was studied using AFM (atomic force microscopy).  Figure 6(a) shows the AFM images of the TiO_2_ nanoparticles, and Figure 6(b) shows the AFM images of the *A. paniculata* plant extract. With increasing temperature, the surface morphology and roughness of TiO_2_ nanoparticles are changed significantly due to phase transformation of anatase to rutile and growth of TiO_2_ crystallites. When compared with the SEM and EDAX analysis, it is observed that no other impurities are present [39].

### 3.7. Thermogravimetric Analysis

Thermal properties of TiO_2_ nanoparticles were studied using thermogravimetric analysis.  Figure 7 shows the TGA curves of TiO_2_ nanoparticles. The graph illustrates weight loss at 40°C due to the release of humidity and organic compounds. The weight loss up to 40°C of the As-prepared sample is approximately 2.387% and was ascribed to desorption of physically adsorbed/retained water and volatility of the alcohol and acetone solvent. The second weight loss between 460°C reflected the elimination of chemically bonded water and the thermal decomposition of organic plant residues [40].

### 3.8. Antibacterial Activity

The antibacterial activity of green synthesized TiO_2_ nanoparticles was carried out by the agar well diffusion method against *Escherichia coli*, *Salmonella* sp., and *Bacillus* sp. The antibacterial activity of TiO_2_ nanoparticles is shown in Figure 8. The high zone of inhibition was observed in *Salmonella* sp., whereas the zone of inhibition for *E. coli* and *Bacillus* sp. was less. It shows that the zone inhibition was increased with the TiO_2_ nanoparticle. The zone of inhibition was measured in mm. Titanium dioxide nanoparticles are effectively involved in the inhibition of bacterial growth [41, 42]. The antifungal activity was tested against *Candida albicans*. It shows that the zone of inhibition was raised and resulted in the green synthesized TiO_2_ nanoparticles antifungal activity against *Candida albicans*.

### 3.9. Antioxidant Activity (DPPH Radical Scavenging)

Figure 9 shows that the synthesized TiO_2_ nanoparticles show the increased concentration of the antioxidant activity. The previous research shows that the antioxidant activity of TiO_2_ nanoparticles has good antioxidant activity. Hence, it is confirmed that the TiO_2_ nanoparticles synthesized using *A. paniculata* also have antioxidant activity. Nowadays, nanoparticles are widely used for antioxidant activity to improve their biomedical applications [43–45].

### 3.10. Antidiabetic Activity

The antidiabetic activity of *A. paniculata*-mediated titanium dioxide nanoparticles was performed using alpha-amylase assay (Figure 10). 10 *μ*L of *α*-amylase solution (0.025 mg/mL) was added with 240 *μ*L of phosphate buffer containing a different concentration of plant extract. Incubate at 37°C. 100 *μ*L of the starch solution was added to the plant extract with 5 ml of distilled water. Blank is taken as without *α* amylase, whereas control is without a starch solution. Absorbance was taken at 565 nm. The antidiabetic activity for the synthesized TiO_2_ nanoparticles shows the increased concentration. To the best of our knowledge, fewer documents are available for the antidiabetic activity of TiO_2_ nanoparticles.

### 3.11. In Vivo Toxicity Green Synthesis of TiO_2_ Nanoparticles

The hatching rates of zebrafish embryos exposed to various concentrations of titanium dioxide nanoparticles at early embryonic stages are shown in Figure 11. During the reasonable condition, zebrafish embryos had a hatching period from 48 to 72 hpf. TiO_2_ particle size is 50 nm, which was less than the size of the chorion; it is 0.5–0.7 *μ*m. This particle size entered the embryos across the chorion via pores [46]. The agglomeration of particles blocks the pores, reducing the exchange of nutrients [47]. However, our particles are not sediment and undergo agglomeration, so they racially transport the nutrient exchange to chorion pores. Compared to the control group, 150 *μ*g/L titanium dioxide nanoparticle-treated groups showed significant hatching delay. However, ≥150 *μ*g/L of *Andrographis paniculata*-mediated titanium dioxide nanoparticle displayed a lack of embryonic hatchability. The embryonic cell cycle at 28–48 hpf retina cells of the inner nuclear layer is postmitotic [48, 49]. This study shows that the nuclear layer begins to differentiate. However, it can be identified at 72 hpf in the photoreceptor region. Our data showed that titanium dioxide exposure caused developmental toxicity and a normal and healthy hatching effect on immature zebrafish embryos.

The embryos were exposed to 0–250 *μ*g of titanium dioxide nanoparticles, and the abnormality was observed at 24–72 hpf, which is shown in Figure 12. However, at a concentration of ≥250 *μ*g/L of titanium dioxide nanoparticles, treated embryos and larvae exhibited acute malformations and unhatched embryos, which had coagulated (Figure 13). At ≥200 *μ*g/L and 250 *μ*g/L concentrations, affected embryos were unable to hatch and eventually died. The exposure of control solutions (E3 medium) to zebrafish embryos did not produce any developmental defects. The titanium dioxide nanoparticle treated group had significantly lesser malformation rates even at the highest concentration. Several malformation patterns, including yolk-sac and pericardial edema tail bent, axis bent, and spinal curvature, have not been observed in the titanium dioxide nanoparticle-treated group as shown in Figure 13. These observations showed that titanium dioxide nanoparticles not induced any embryonic phenotype on developing embryos. In a previous study, titanium dioxide nanoparticles were green synthesized using *Sesbania grandiflora* leaf extract, and the results showed a higher malformation rate in 48–72 hpf zebrafish embryos at the highest concentration of 2.5 mg/L [50]. The current study results proved that *Andrographis paniculata* leaf extract-mediated titanium dioxide nanoparticles at the lowest concentration (250 *μ*g/L) does not cause any malformation in zebrafish embryos.

## 4. Conclusions

Phytosynthesized TiO_2_ NPs from the leaf extract of *A. paniculata* has ecofriendly and low-cost material from a plant source. The synthesized material can serve a high quantity of industrial production using biodegradable and reusable natural resources. The presence and character of TiO_2_ NPs confirmed by XRD, SEM, EDX, AFM, TEM, and TGA and in a dose-dependent approach, like antibacterial activity, would reduce pathogenic microorganisms such as *E. coli*, *Bacillus* sp., and *Salmonella typhi* and fungus-like *C. albicans* significant of medical applications. TiO_2_ NPs had a significant impact on the surface of the embryo. The green synthesized TiO_2_ NPs using *A. paniculata* leaf extract showed the potential toxicity for zebrafish.

## Figures and Tables

**Figure 1:** Visual observation of (a) *A. paniculata* plant extract (b) and synthesized TiO_2_ NPs.

**Figure 2:** UV-Vis spectroscopic analysis of TiO_2_ NPs by *A. paniculata*.

**Figure 3:** (a) SEM used shape of particle and (b) EDX used element of TiO_2_ NPs by *A. paniculata* nanoparticle.

**Figure 4:** (a) HRTEM used size of image and (b) DLS used stable of TiO_2_ NPs by *A. paniculata* nanoparticle.

**Figure 5:** XRD analysis of TiO_2_ NPs by *A. paniculata*.

**Figure 6:** AFM analysis of (a) TiO_2_ (b) and *A. paniculata* plant extract.

**Figure 7:** TGA analysis of TiO_2_ NPs.

**Figure 8:** Antibacterial activity of TiO_2_ NPs by *A. paniculata* and its mechanism of action.

**Figure 9:** Antioxidant activity of TiO_2_ NPs by *A. paniculata*.

**Figure 10:** Antidiabetic activity of TiO_2_ NPs by *A. paniculata*.

**Figure 11:** Hatching rate of the zebrafish embryos treated with TiO_2_ nanoparticles.

**Figure 12:** Viability rate of the zebrafish embryos treated with TiO_2_ nanoparticles.

**Figure 13:** Zebrafish embryo hatching, viability, and hatching delay in zebrafish embryos.

## Data Availability

The data used to support the findings of this study are included within the article.
